# Clinical Utility of the Prenatal Ultrasound Score of the Placenta Combined with Magnetic Resonance Imaging in Diagnosis of Placenta Accreta during the Second and Third Trimester of Pregnancy

**DOI:** 10.1155/2022/9462139

**Published:** 2022-06-15

**Authors:** Jing Zhang, Pingping Dong

**Affiliations:** ^1^Department of Ultrasonography, Wuhan Hankou Hospital, Wuhan 430012, Hubei, China; ^2^Department of Obstetrics, Yantai Mountain Hospital, Yantai 264001, Shandong, China

## Abstract

**Objective:**

The aim is to explore the clinical utility of the prenatal ultrasound score of the placenta combined with magnetic resonance imaging (MRI) in diagnosis of placenta accreta during the second and third trimester of pregnancy.

**Materials and Methods:**

A total of 108 pregnant women with suspected placenta accreta treated in Wuhan Hankou Hospital and Yantaishan Hospital of Yantai from January 2019 to January 2022 were retrospectively analyzed, the enrolled pregnant women received MRI examination because of suspected results of ultrasonic diagnosis, and by taking pathologic findings as the gold standard, the diagnostic efficacy of the ultrasound score, MRI, and their combination to placenta accreta during the second and third trimester of pregnancy was analyzed, and the diagnostic sensitivity, specificity, the positive predictive value, and the negative predictive value of these diagnostic modalities were evaluated.

**Results:**

Among 108 patients with suspected placenta accreta, 75 with pathologically confirmed placenta accreta were included in the accreta group, and 33 without placenta accreta were included in the non-accreta group; no statistical between-group differences in the patients' age, gestational weeks, educational degree, and other general data were observed (*P* > 0.05), but the history of cesarean section, history of induced abortion, and incidence rate of placenta praevia were significantly higher in the accreta group than in the non-accreta group (*P* < 0.05); the ultrasound score was significantly higher in the accreta group than in the non-accreta group (*P* < 0.05); the incidence rates of signs of “placental heterogeneity” and “bulge of lower segment of the uterus and local thickening of the placenta” were obviously higher in the accreta group than in the non-accreta group (*P* < 0.05); according to the comparison with pathologic findings, the accuracy rate, sensitivity, specificity, the positive predictive value, and the negative predictive value of combined diagnosis were significantly higher than those of single application of the ultrasound score and MRI diagnosis (*P* < 0.05); and ROC analysis found that the area under the curve of combined diagnosis was obviously larger than that of the ultrasound score and MRI diagnosis (*P* < 0.05).

**Conclusion:**

A combining prenatal ultrasound score of the placenta with MRI plays an important role in the diagnosis of placenta accreta during the second and third trimester of pregnancy, which can further improve the diagnostic accuracy rate of placenta accreta and provide significant guidance in preventing high-risk complications during the perinatal period.

## 1. Introduction

Placenta accreta refers to a disease and critical obstetric complication in which placental tissue invades the myometrium to varying degrees, which manifests as the failure of natural separation of some or all of the placenta after delivery, and may lead to severe postpartum hemorrhage and shock. According to epidemiological investigation and statistics, the incidence rate of placenta accreta has increased nearly 20 times in recent years, and the disease has become an important cause of postpartum hemorrhage, perinatal emergency hysterectomy, and maternal death [1, 2]. Therefore, prenatal accurate diagnosis of the placental situation is essential to ensure life safety for both the mother and fetus before delivery and is highly instructive to clinically develop treatment schemes and avoid the risk of multiple complications. Recently, medical imaging examination is becoming more and more important in clinical work, especially magnetic resonance imaging (MRI) examination, which has advantages irreplaceable by other imaging examinations in the localization and qualitative diagnosis of lesions [3, 4]. Currently, the two most commonly used methods for diagnosis of placenta accreta are ultrasound and MRI, and ultrasound is considered to be the preferred method because of its low cost, noninvasiveness, and simplicity of operation, which is able to determine the location and predict the status of placenta accreta [5, 6]. However, ultrasound is easily affected by operator technique, placental location, the amount of amniotic fluid, the thicker adipose tissue in the abdominal wall of pregnant women, and other factors that lead to unclear visualization of the placenta on the back wall of the uterus, and thus has some limitations. MRI, with high soft tissue resolution, no ionizing radiation, multi-directional imaging, and large scanning field, together with the recent development of rapid scanning technology and image processing methods, better solves the problem of fetal movement artifacts, making it increasingly advantageous in fetal examination and becoming another important examination after ultrasound examination for the diagnosis of obstetric diseases [7]. Therefore, ultrasound combined with MRI has a high potential application in the diagnosis of placenta accreta. Besides, due to varied study designs and evaluation methods, the accuracy rates of ultrasound and MRI in diagnosing placenta accreta were not the same in different published works. Based on this, the clinical utility of the prenatal ultrasound score of the placenta combined with MRI in the diagnosis of placenta accreta during the second and third trimester of pregnancy was explored herein, in the hope of providing a reference for clinical prognosis and condition evaluation.

## 2. Materials and Methods

### 2.1. Inclusion Criteria

Inclusion criteria were as follows: (1) All patients received ultrasound and MRI examinations and had no corresponding contraindications; (2) patients were at least 20 years old; (3) patients were pregnant with only one baby at a time; (4) the gestational age of pregnant women were not less than 28 weeks; and (5) patients and their family members understood the study objective and process, and signed informed consent.

### 2.2. Exclusion Criteria

Exclusion criteria were as follows: (1) Patients were complicated with severe liver and kidney dysfunction, malignant tumor, or coagulation dysfunction; (2) patients had other pregnancy complications, such as gestational hypertension and gestational diabetes mellitus; (3) patients had cognitive disorder, verbal communication disorder, or limb movement disorder; and (4) patients had lower compliance and incomplete clinical data.

### 2.3. Screening and Grouping of Patients

A total of 108 pregnant women with suspected placenta accreta treated in Wuhan Hankou Hospital and Yantaishan Hospital of Yantai from January 2019 to January 2022 were screened for the retrospective analysis study and, respectively, included in the accreta group and the non-accreta group according to their final pathologic findings. The study plan met the ethnic and moral code and the World Medical Association Declaration of Helsinki (2013) [8], and was reviewed and approved by the Ethics Committee of Wuhan Hankou Hospital and Yantaishan Hospital of Yantai.

### 2.4. Methods

#### 2.4.1. Ultrasound Examination

The ultrasound examination was conducted to patients by the ultrasonic diagnostic apparatus (Siemens Acuson S2000 and Philips Affiniti 70), the frequency of the abdominal probe was set as 2–7 MHz, and the frequency of the transvaginal probe was set as 4–9 MHz. Pregnant women were in the conventional supine position and took the lateral recumbent position, when necessary, with filling of the bladder before examination. The conventional ultrasound examination by abdomen was conducted first, the comprehensive two-dimensional and color Doppler scan was performed on the vertical section, cross-section, and crown section of the placental attachment range, and if the ultrasound examination by the abdomen failed to obtain the desirable effect or placenta accreta was suspected; then, a transvaginal scan was performed [7]. Finally, scores were given according to the patients' ultrasonic characteristics to evaluate the degree of placenta accreta.

#### 2.4.2. MRI Examination

The 1.5 T superconducting MRI diagnostic apparatus (model: Siemens Avanto; manufacturer: Siemens AG) and the abdominal phased array coil were used for the examination of patients. Before examination, pregnant women were warned repeatedly to appropriately hold back urine to clearly show the bottom of the bladder. The supine position was taken, head first or foot first was selected according to the actual situation of pregnant women, and scanning was performed from pubic symphysis to the superior edge of the placenta. The sequences were set as follows. T_1_WI cross-section (turbo spin echo (TSE)) T_1_WI: FOV 400 × 360 mm, TR 560 ms, TE 9 ms, 2 mm slice interval, 6 mm slice thickness, matrix 256 × 256, flip angle 150°, and 35 slices scanned; T_2_WI cross-section, sagittal position, and coronal position, half-Fourier acquisition single-shot turbo spin-echo (HASTE) T_2_WI: FOV 400 × 400 mm, TR 1,200 ms, TE 60 ms, 0 slice interval, 6-7 mm slice thickness, matrix 256 × 256, flip angle 150°, and 35 slices scanned.

### 2.5. Diagnostic Criteria

#### 2.5.1. Surgical Pathological Diagnosis

Placenta accreta. The continuity of the muscular layer under the surface of placental attachment was interrupted, local or all muscular layer structure disappeared and only the serosal layer was found, placental attachment could be seen through the serosal surface, the separation surface was massively bleeding which was not easily controlled by uterotonic drugs, and uterine pathological findings revealed invasion of the villus structure into the muscular layer.

No placenta accreta. The myometrium at the surface of placental attachment was intact, the placenta could be separated free by itself or manually, the placenta and the uterus were easily separated without obstructing sensation, the separated surface was smooth and complete without major bleeding points or with only a small amount of oozing blood.

#### 2.5.2. Ultrasound Scores

Scores were given according to the placenta location, thickness, postplacental low echo band, bladder line, placental lacunae, blood flow signals at the base of the placenta, cervical sinusoid, cervical morphology, and history of cesarean section. Specific scoring criteria is shown in Table 1 [9].

#### 2.5.3. MRI Examination

No less than two senior physicians read the images and made MRI imaging diagnoses, and in case of diagnostic disagreement, repeat reading was required until consensus was reached; MRI diagnostic criteria were divided into direct signs and indirect signs with reference to the relevant literature [10].

Direct signs of placenta accreta are as follows: disappearance of the utero-placental interface, interruption of the myometrial signal, invasion of the placental tissue signal into the myometrial or parametrial tissue, and viscera.

Indirect signs of placenta accreta are as follows: (1) placental heterogeneity, indicated by the presence of intraplacental banded hypointensity on the T_2_WI sequence; (2) unclear boundaries on the placenta-myometrium interface; (3) the lower segment of the uterus was bulging outward, and the local placenta was markedly thickened; (4) placental vessels were thickened and increased; (5) the bladder showed locally “tent”-like change or nodular projections. The indirect signs of placenta accreta in pregnant women were mainly observed in this study.

### 2.6. Statistical Processing

The between-group differences in the data obtained in the study were calculated by the SPSS22.0 software, the items included were enumeration data and measurement data, which were expressed by [*n*(%)] and ($\bar{\text{x}}$ ± *s*) and examined by the *X*^2^ test and the *t*-test, respectively, and differences were considered statistically significant at *P* < 0.05.

## 3. Results

### 3.1. Results of Pathological Diagnosis

Among 108 patients with suspected placenta accreta, 75 with pathologically confirmed placenta accreta were included in the accreta group, and 33 without placenta accreta were included in the non-accreta group; no statistical between-group differences in the patients' age, gestational weeks, educational degree, and other general data were observed (*P* > 0.05), but the history of cesarean section, history of induced abortion, and incidence rate of placenta praevia were significantly higher in the accreta group than in the non-accreta group (*P* < 0.05) (see Table 2).

### 3.2. Ultrasound Score Diagnosis

The statistics in Table 3 showed that the ultrasound score of the accreta group was significantly higher than that of the non-accreta group (*P* < 0.05), indicating statistically significant difference.

### 3.3. MRI Signs

Table 4 showed that the incidence rates of signs of “placental heterogeneity” and “bulge of lower segment of the uterus and local thickening of the placenta” were obviously higher in the accreta group than in the non-accreta group (*P* < 0.05).

### 3.4. Diagnostic Efficacy

According to the comparison with pathologic findings, the accuracy rate, sensitivity, specificity, the positive predictive value, and the negative predictive value of combined diagnosis were significantly higher than those of single application of the ultrasound score and MRI diagnosis (*P* < 0.05); and ROC analysis found that the area under the curve of combined diagnosis was obviously larger than that of the ultrasound score and MRI diagnosis (*P* < 0.05) (see Tables 5 and 6, Figure 1, and Table 7).

## 4. Discussion

Placenta accreta is an abnormal placenta implantation due to congenital aplasia of the endometrium or traumatic endometrial defect, incomplete decidualization of the endometrium at the defect during the first trimester, and invasion or penetration of the myometrium by placental villous tissue from the defect, which is often accompanied by placenta praevia, can cause major maternal hemorrhage, has a high lethality rate, and is one of the serious obstetric complications, seriously threatening the life safety of both mother and fetus [11]. Generally, when the placental villus erodes and implants into the endometrium, decidual tissue has a certain barrier protective effect against villus invasion, and thus the occurrence of placental accreta depends on the balance between the implantation force of placental villous tissue and decidual tissue against villus erosion, and once such balance is broken, villous tissue with high invasive ability is able to invade or penetrate the myometrium through the defective decidua and then form pathological placental accreta. By conducting analysis from a theoretical point of view, it is found that factors capable of triggering primary decidual dysgenesis or secondary endometrial damage, such as adenomyosis, uterine malformation, induced abortion, and endometrial infection, may cause placenta accreta. Based on the findings of relevant studies at home and abroad [12–14], it is generally believed that advanced maternal age, cesarean delivery, induced abortion, placenta praevia, and history of uterine surgery are high-risk factors for triggering placenta accreta, of which placenta praevia and cesarean delivery are the most significant, while advanced maternal age and placenta praevia are considered to be two independent risk factors for placenta accreta. Among 108 patients with suspected placenta accreta, 75 with pathologically confirmed placenta accreta were included in the accreta group, and 33 without placenta accreta were included in the non-accreta group; no statistical between-group differences in patients' age, gestational weeks, educational degree, and other general data were observed (*P* > 0.05), but the history of cesarean section, history of induced abortion, and the incidence rate of placenta praevia were significantly higher in the accreta group than in the non-accreta group (*P* < 0.05). The results were consistent with the previous studies[15–17], which considered that placenta accreta is strongly associated with cesarean delivery, induced abortion, and placenta praevia. The occurrence of placenta praevia is mainly due to abnormal placental villus implantation during the first trimester of pregnancy that limits the ability of the placenta to move up with the enlarged uterus. The subjects of this study were all suspected of having placenta accreta and had a higher probability of placenta praevia. The selection of subjects may be biased, and thus placenta accreta and the presentation of placenta praevia are highly correlated. According to related findings [18, 19], nowadays, with the opening of China's fertility policy, the social pressure on women increases, resulting in higher childbearing age of women, and many studies have shown that the incidence of placenta accreta will increase with maternal age. Although the proportion of patients aged >35 years in the accreta group was higher than that in the non-accreta group in this study, the difference was not significant, which may be due to the small sample size, so an in-depth study with an expanded sample size should be carried out.

Analysis on the patients' prenatal ultrasound score of the placenta found that the score was significantly higher in the accreta group than in the non-accreta group (*P* < 0.05), which confirmed that it was feasible for the prenatal ultrasound score of the placenta to diagnose placenta accreta with multiple ultrasound signs. The placental ultrasound score mainly assesses patients for high-risk factors around the uterine thickness of the thinnest part, number of cesarean sections and deliveries, placental lacunae, and border-crossing vessels, which is beneficial for individualized prenatal risk stratification and assessment and providing a basis for treatment options and planned delivery. The subjects of this study were mainly patients in the second and third trimester who had a thinner myometrium and increased placental folds with insignificant direct signs, and even direct signs are observed, it is difficult to make an accurate judgment, thus indirect signs of placental accreta observation is particularly important for patient diagnosis. The study results showed that the incidence rates of signs of “placental heterogeneity” and “bulge of lower segment of the uterus and local thickening of the placenta” were obviously higher in the accreta group than in the non-accreta group (*P* < 0.05), which was consistent with the previous study [20]. “Placental heterogeneity” is a lesion showed low iso-intensity signals on T_1_WI, which is considered the most characteristic and a sensitive sign; “bulge of lower segment of the uterus and local thickening of the placenta” also present a higher diagnostic value for placenta accreta, and can be used jointly with “placental heterogeneity” to improve the diagnostic accuracy rate of placenta accreta. According to the comparison with pathologic findings, the accuracy rate, sensitivity, specificity, the positive predictive value, and the negative predictive value of combined diagnosis were significantly higher than those of single application of the ultrasound score and MRI diagnosis (*P* < 0.05); and ROC analysis found that the area under the curve of combined diagnosis was obviously larger than that of the ultrasound score and MRI diagnosis (*P* < 0.05), demonstrating that the results of the combining prenatal ultrasound score of the placenta with MRI diagnosis were highly consistent with pathologic findings, presenting a high diagnostic accuracy rate, and that combined diagnosis had higher sensitivity and specificity than single examination.

Ultrasonic testing has the advantages of easy operation, high safety and noninvasiveness, real-time imaging, and reproducible examination, and has the ability to observe the blood flow situation while examining the placenta, so it is indispensable and important in obstetric clinical diagnosis [21, 22]. However, the affecting factors of ultrasound examination, such as maternal body type, bone, and intestinal gas, easily reduce the penetration of the ultrasonic wave or increase the reflection wave, leading to poor observation at the pathogenic lesion and declined ability to observe lesions on the posterior uterine wall, and thus placenta accreta in the posterior uterine wall is a blind area for ultrasound examination. However, MRI examination of soft tissue with high contrast and wide view is able to acquire the anatomical relationship of intact placental tissue and surrounding structures, and the adverse factors of ultrasound, such as maternal body type, bone, and intestinal gas, have less influence on MRI, and therefore, even when there is less amniotic fluid or the placenta is located in the posterior wall of the uterus, MRI examination can still provide a clear and accurate image and perfectly show the location and morphology of placenta accreta, making it a significant prenatal imaging modality for the diagnosis of placenta accreta besides ultrasound examination [23–25]. In addition, the sample size of this study was relatively small, which still needs to be supported by data from a large sample study. It was a retrospective study with the advantage that the conditions were less restrictive, but the patients' current physical and mental status may affect the authenticity and accuracy of past data.

In conclusion, combining prenatal ultrasound score of placenta with MRI plays an important role in the diagnosis of placenta accreta during the second and third trimester of pregnancy, which can promote the contrast between placenta and uterus, help to distinguish and judge the relationship between the two and accurately determine the pathological pattern of placenta accreta before delivery, and promote the diagnostic accuracy rate of placenta accreta. Therefore, such modality is highly instructive for preventing high-risk complications during the perinatal period. For patients meeting the examination indications, the combined examination should be recommended.

## Figures and Tables

**Figure 1:** ROC curve.

**Table 1:** Ultrasound scoring criteria for placenta accreta.

Evaluation dimension	2 points	1 point	0 point
Placenta location	Complete praevia	Marginal or low-lying	Normal
Placenta thickness	>5 cm	3–5 cm	<3 cm
Postplacental low echo band	Disappeared	Locally interrupted	Continuous
Bladder line	Disappeared	Interrupted	Continuous
Placental lacunae	Fused into patch	Yes	No
Blood flow signals at the base of the placenta	Appearance of “border-crossing” blood vessel	Increasing or agglomerating blood flow	Regular basilar blood flow
Cervical sinusoid	Fused into patch	Yes	No
Cervical morphology	Disappeared	Not complete	Complete
History of caesarean section	Twice and above	Once	No

**Table 2:** Between-group comparison of patients' general data.

Observation indicator	Accreta group (*n* = 75)	Non-accreta group (*n* = 33)	*X* ^2^/*t*	*P*
Age (years)			1.767	0.184
≥35 years	28 (37.33%)	8 (24.24%)		
<35 years	47 (62.67%)	25 (75.76%)		
Gestational age (weeks)	32.67 ± 2.69	32.88 ± 2.46	0.383	0.702
History of cesarean section	31 (41.33%)	7 (21.21%)	4.068	0.044
History of induced abortion	36 (48.00%)	9 (27.27%)	4.051	0.044
Placenta praevia	60 (80.00%)	19 (57.58%)	5.867	0.015
Educational degree			0.019	0.892
Senior high school and below	24 (32.00%)	11 (33.33%)		
Senior high school and above	51 (68.00%)	22 (66.67%)		

**Table 3:** Between-group comparison of ultrasound scores.

Group	Number of cases	Ultrasound score
Accreta group	75	8.05 ± 1.52
Non-accreta group	33	1.94 ± 0.74
*t*		21.934
*P*		<0.001

**Table 4:** Between-group comparison of patients' MRI signs [*n*(%)].

MRI signs	Accreta group (*n* = 75)	Non-accreta group (*n* = 33)	*X* ^2^	*P*
Placental heterogeneity	39 (52)	4 (12.12)	15.209	<0.001
Non-distinct placenta-uterus boundary	35 (46.67)	14 (42.42)	0.166	0.683
Bulge of lower segment of the uterus and local thickening of the placenta	37 (49.33)	2 (6.06)	18.600	<0.001
Increased local blood vessel in the placenta	33 (44)	12 (36.36)	0.550	0.458
Local tentiform thickening or nodular projection of the bladder	19 (25.33)	5 (15.15)	1.375	0.241

**Table 5:** Comparison with pathologic findings.

Pathologic findings	Ultrasound score		MRI		Combined diagnosis		Total
	Accreta	Non-accreta	Accreta	Non-accreta	Accreta	Non-accreta	
Accreta	66	9	69	6	71	4	75
Non-accreta	11	22	9	24	4	29	33
Total	77	31	78	30	75	33	

**Table 6:** Diagnostic efficacy (%).

Test variable	Accuracy rate	Sensitivity	Specificity	Positive predictive value	Negative predictive value
Ultrasound score	81.48^*∗*^	88.00^*∗*^	66.67^*∗*^	85.71^*∗*^	70.97^*∗*^
MRI	86.11^*∗*^	92.00^*∗*^	72.73^*∗*^	88.46^*∗*^	80.00^*∗*^
Combined diagnosis	92.59	94.67	87.88	94.67	87.88

*Note.* sensitivity = number of positive cases/total number of cases; specificity = number of negative cases/total number of cases; accuracy rate = number of accurately diagnosed cases/total number of cases; positive predictive value = number of false positive cases/total number of positive cases; negative predictive value = number of false negative cases/total number of negative cases; ^*∗*^ indicated statistically significant difference when comparing with combined diagnosis (*P* < 0.05).

**Table 7:** Area under the curve.

Test result variable	Area	Standard error a	Asymptotic Sig b	Asymptotic 95% confidence interval
Ultrasound score	0.773	0.054	0.000	0.668–0.879
MRI	0.824	0.050	0.000	0.726–0.921
Combined diagnosis	0.913	0.036	0.000	0.841–0.984

*Note.* a. under nonparametric assumptions; b. null hypothesis: real area = 0.5; Sig b indicated significance.

## Data Availability

Data that support the findings of this study are available on reasonable request from the corresponding author.
